The article "Research on the Implementation Path of Ideological and Political Education in Private Colleges and Universities under the Network Environment" was retracted in 2023. Reasons: signs of a paper mill; suspected computer-generated content; unreliable results or conclusions; lack of ethics approval or compliance.

# Research on the Implementation Path of Ideological and Political Education in Private Colleges and Universities under the Network Environment

**DOI:** 10.1155/2022/2830388

**Published:** 2022-07-12

**Authors:** Da Luo

**Affiliations:** Software Engineering Institute, Guangzhou 510990, China

## Abstract

Entering the network information age, all kinds of excellent and backward ideas and value orientations coexist on the network, and social trends of thought are diverse. Therefore, colleges and universities need to occupy the network position, expand the educational position from the platform to the network world, and better lead the Ideological and Political Education (IPE) of college students. Therefore, this paper takes the practice of IPE in China's Private Colleges and Universities (PCU) under the network environment as the research object. Firstly, this paper expounds the definition of PCU and briefly introduces the basic theory of IPE of college students. Secondly, it investigates the current situation of students' IPE under the network environment and analyzes the implementation path. Finally, through research and argumentation, the current situation and influencing factors of IPE in PCU are clarified, and countermeasures and suggestions are provided for online teaching in universities.

## 1. Introduction

PCU shoulder the important mission of educating talents for the country and the party together with public colleges and universities [1]. Network IPE has become the most important in PCU [2]. College students, as the new people of the times, the party, and the state have the inescapable responsibility and obligation to IPE of college students. In the late 1990s, scholar Zhang Jiansong [3] proposed that “the network ideological and political work of PCU actually implements ideological and political work on students through the campus network.”

Nowadays, the living environment of college students is much richer than that of primary and secondary school students. Born as a person, the perception of natural environment and social environment will affect every student's thoughts and values. If we want to establish correct values and outlook on life, we must carefully perceive all the surrounding environments. From a philosophical point of view, the influence of environment on human thought is ubiquitous. In order to deliver better ideological and political courses to college students and guide them to correctly perceive nature and the environment, it is essential to proceed education reform.

“Online learning” is a method of learning through the Internet without any restrictions on location [4]. During the epidemic period, online teaching has been widely used to achieve normal teaching tasks under the premise of safety [5]. IPE courses also quickly set up online classes, timely propaganda of epidemic prevention, and control knowledge. Interpret the spirit of the important instructions of the government in epidemic prevention and control work from multiple perspectives and levels, and actively publicize the story of fighting the epidemic.

The article "Research on the Implementation Path of Ideological and Political Education in Private Colleges and Universities under the Network Environment" was retracted in 2023. Reasons: signs of a paper mill; suspected computer-generated content; unreliable results or conclusions; lack of ethics approval or compliance.

The development of IPE needs to rely on the orientation of the times, grasp the “times, moderate, effective,” and further construct a more targeted and contemporary theoretical and practical system [6]. On the other hand, network technology needs to be combined with the traditional advantages of IPE to become the new vitality of education [7]. The following is the number of Chinese Internet users according to official data (see Figure 1).

From Figures 2 and 3, it is not difficult to find that in 2016, the age group of Internet users in Internet penetration rate is 20 to 29 years old, accounting for 30.5%. In terms of education level, the highest percentage of Internet users is middle school and above, accounting for 85%.

Through data analysis, it is not difficult to find that most groups using the Internet are young people, and most of them have received secondary education or above. Therefore, it is important to study the practical path of IPE in China.

The innovations of this paper are as follows:

1. It expounds the definition of private colleges and universities and briefly introduces the basic theory of ideological and political education of college students.
2. It investigates the current situation of students' ideological and political education under the network environment and analyzes the implementation path.
3. It clarifies the current situation and influencing factors of IPE in PCU and provides countermeasures and suggestions for online teaching in colleges and universities

This paper consists of five main parts: the first part is the introduction, the second part is state of the art, the third part is the methodology, the fourth part is the result analysis and discussion, and the fifth part is the conclusion.

## 2. State of the Art

The first official document put forward by PCU in China is the Interim Provisions on the establishment of PCU, which was issued in 1993 [8]. PCU refer to various social organizations and individual citizens other than state organs and state-owned enterprises and institutions, which raise their own funds and set up higher academic education institutions in accordance with the provisions. According to the regulations, the schools funded by domestic social organizations and individuals that are not national institutions in China are called “private schools,” and the education carried out is called “private education.” According to the students' age and academic background, private education in China can be divided into six categories: private preschool, private compulsory, private high school, private secondary vocational, private colleges, and training institutions. The private education mentioned in this study is all private higher education except for special reference. The “Private Education Promotion Law” issued that private education is also public welfare education, equal to public education. In China, universities are usually divided into two types: general higher education schools and private general higher education schools (i.e., PCU) [9].

The article "Research on the Implementation Path of Ideological and Political Education in Private Colleges and Universities under the Network Environment" was retracted in 2023. Reasons: signs of a paper mill; suspected computer-generated content; unreliable results or conclusions; lack of ethics approval or compliance.

In this study, the definition of “ideological and political education” refers to the comprehensive education implementation process of comprehensive participation and implementation for college students through curriculum education, network education, and other comprehensive education systems [10].

The academic circle has a relatively unified interpretation of “IPE,” which is put forward by a scholar. “IPE refers to the purposeful, planned, and organized influence exerted by a society or social group on its members with certain ideological concepts, political viewpoints, and moral norms [11] so that they can form social practice activities that meet the ideological and moral needs of a certain society and a certain class.”

Nowadays, the Internet has become indispensable in the student groups of PCU in China, and the influence has also begun to be paid attention to.

Network education students are educated, the teacher is the educator, under the help and guidance of educators, through the network to learn [12]. Network provides advanced teaching methods and rich teaching content, which is a brand-new education model. Its main characteristic is to rely on the network technology as a teaching method, on the Internet directly transregional a new interactive teaching mode. Modern distance education also relies on the network to achieve better benefit.

As for the definition of network IPE, many scholars have put forward their own views from their own perspectives [13]. The definition given by scholar Liu Mei [14] is that “network IPE is a new theory to realize ideological propaganda based on the theory of communication and realize the purpose of education through network technology.” This is the earliest definition elaboration in our country. In fact, there is a partial problem in the explanation of this concept. It does not give real-time guidance to people who use the network but explains how to use the network in the way of using tools. Therefore, this concept cannot be completely generalized. In recent years, China has begun to attach importance to this field, and many scholars have also begun to devote their energy to research. Scholar Yang Liying [15] believes that “Network IPE firstly takes the network as the carrier and uses communication and ideological propaganda theories to carry out education, which has become a mode of IPE adapted to the contemporary era.” A scholar [16] also gave his own view: “to realize network ideological and political education, we must grasp the internal characteristics of the network and make a large-scale and planned impact on college students' IPE and moral norms through the network so as to make their morality meet the social needs.” In short, many scholars have given their own opinions on the connotation of IPE for college students from different heights, which also provides a direction for PCU to fully understand the nature of IPE for college students under the network environment.

The article "Research on the Implementation Path of Ideological and Political Education in Private Colleges and Universities under the Network Environment" was retracted in 2023. Reasons: signs of a paper mill; suspected computer-generated content; unreliable results or conclusions; lack of ethics approval or compliance.

## 3. Methodology

### 3.1. The Current Situation of Internet Information Use among Contemporary Students

More than 90% of Chinese college students surf the Internet, and nearly 50% of them surf the Internet frequently [17]. Therefore, we can see that the Internet has gradually entered into people's daily life, from value orientation to behavior mode, from moral thought to psychological development, it brought a huge impact on students' daily life.

Universities are the experiencer and promoter of informatization tide, and the development frontier of “network” in our society. It has become an urgent problem to explore how to strengthen the IPE of college students under the network environment [18]. The age distribution and education level of Chinese netizens are shown in Figures 4 and 5.

As can be seen from the graph above, the group between the ages of 18 and 29 accounts for the highest proportion of Internet users. Among Internet users, those with college degree or above account for 47.1%. College students, as the elites of the times, are also the forefront of Internet use and shoulder heavier social responsibilities than other groups.

Because of the emergence of the network, college students' learning knowledge is no longer confined to textbooks or the teaching of educators in the classroom. With the Internet as a platform, a variety of rich knowledge and information into the eyes of college students, college students can be 24/7 nonstop learning. People can learn about the world and get information through the Internet anytime and anywhere. According to a survey, most college students believe that the Internet is helpful for their professional learning (see Table 1).

The article "Research on the Implementation Path of Ideological and Political Education in Private Colleges and Universities under the Network Environment" was retracted in 2023. Reasons: signs of a paper mill; suspected computer-generated content; unreliable results or conclusions; lack of ethics approval or compliance.

The Internet itself is open, which makes traditional spatial boundaries disappear and makes real-time interaction between people in distant places a real thing. With the increasingly fierce social competition, college students are facing pressure from all aspects. Surfing the Internet is an important part of their choice as a way to relieve stress. In this way, they can expose their feelings to people they know or do not know, vent their emotions, and let the pressure off. Ideological workers can also rely on the Internet to help students solve difficult problems, build up their self-confidence, and prevent tragedies. Through the investigation, it is found that the use of network can have a positive impact on the interpersonal communication mode of college students and also can enrich the form of interpersonal communication and expand the space of interpersonal communication.  Table 2 lists the parameters.

The network has brought college students a brand-new experience, which even exceeds the height and depth they cannot reach in the real world, which makes some weak-willed college students addicted to the illusory network world and unable to extricate themselves. According to the survey, almost 80 percent of the respondents tend to rely on the Internet. And students who are obsessed with the Internet are more likely to develop character defects than those who use the Internet properly. Some even reach the level of Internet addiction and live in their own world all the time. Most college students and teenagers have serious Internet addiction. The report data are shown in Table 3. Many college students say that they feel uncomfortable if they do not surf the Internet every day. Table 3 lists the parameters.

### 3.2. Investigation and Analysis of the Situation of IPE Network Application in Students

“No investigation, no right to speak.” Only by actual investigation, we can deeply understand the application effect of network carrier in college students' IPE [19].

College students have the most say on the application and effect of network carrier. This survey selected a domestic university as the key survey object and combined with the network questionnaire “Survey on the Current Situation of the Application of Network Carrier of Ideological and Political Education for College Students.” The respondents included junior college students, undergraduates, and some postgraduates, among which male and female accounted for 27.75% and 72.25%, respectively. According to educational background, junior college students accounted for 4%, undergraduate students accounted for 49%, and master's degree or above accounted for 47%. By major, 35.25 percent of students majored in literature, history, and philosophy, 41 percent in science and engineering, and 23.75 percent in economics, management, art and sports, medicine, and law. The subjects involved in the investigation process cover a relatively complete range of grades and majors. After comprehensive investigation, the obtained data can truly reflect the real problems.

The article "Research on the Implementation Path of Ideological and Political Education in Private Colleges and Universities under the Network Environment" was retracted in 2023. Reasons: signs of a paper mill; suspected computer-generated content; unreliable results or conclusions; lack of ethics approval or compliance.

The questionnaire involved 30 topics, including single choice, multiple choice, and question and answer questions, covering the development and application of network carrier of IPE for students, their participation, optimization suggestions, and other aspects [20]. It can basically reflect the application status of the network carrier of IPE for college students and help us make further analysis and adjustment.

In the survey, about the question “how do you think the application effect of IPE network carrier?” nearly 90% of the respondents are optimistic about the application effect of IPE network carrier, as shown in Figure 6. 41% think its form is new and more attractive. 16% said it enhanced interaction. Those who think the network carrier is more interesting than the traditional classroom account for 20%. 12.5% thought that the network carrier improved the efficiency of IPE.

First, part of the educators use network carrier proficiency is not high enough. “There is a deep generational gap in the information society, and while children dominate the world's information resources, adults need to work hard and catch up, especially educators.” Educators should first understand the network themselves, have enough understanding of the importance of the network carrier and its unique advantages, and learn to use the network to deeply integrate the network and. Most educators have used the network carrier in educational activities, but some educators still do not want to use the network carrier, do not use, are even suspicious of the attitude of the network carrier, and so on. In addition, some educators are not familiar with the operation of network carriers. Regarding this question in the questionnaire, more than 50% of the respondents think that the proficiency level of educators in using network carriers is not high enough, as shown in Figure 7.

The network carrier not only needs to be used, but also needs to be used effectively. It depends on whether the educator can use the network carrier to communicate deeply with the recipient and enhance the interaction. In the survey results, the frequency of communication between teachers and counsellors and college students through online platforms is discussed. As shown in Figure 8, the proportion of those who think little communication is more than 50%, indicating that the utilization rate of network carrier is not high among educators. Nowadays, almost every college student has a smartphone and a computer, and the Internet goes hand in hand with college students.

The article "Research on the Implementation Path of Ideological and Political Education in Private Colleges and Universities under the Network Environment" was retracted in 2023. Reasons: signs of a paper mill; suspected computer-generated content; unreliable results or conclusions; lack of ethics approval or compliance.

Secondly, some college students have insufficient subjectivity in using the network carrier. Only by fully stimulating the subjectivity and creativity of college students in the use of network carrier can the educational effect of network carrier be effectively brought into play. The survey results show that nearly 90% of college students spend more than three hours on the Internet every day, of which more than 60% spend chatting, watching videos, and listening to music. The main channel for them to obtain information is ideological and political theory courses, as shown in Table 4. These data show that college students have not fully accepted the network as the carrier of IPE.

Thirdly, the network carrier content design is not scientific enough. Under the network environment information unblocked channel height, height of resources sharing for educators to integrate education resources rich education content provides favorable conditions, but the network information is complex, spread more disorderly, need educators according to high education purpose design thoughtful, good fun, wide adaptability, can be both informative and thoughtful information repository. Cognitive psychology and communication studies show that, faced with a variety of information, communication objects only select what they think needs to be recognized, and abandon other irrelevant information. For college students, what they need is information with truth, authenticity, value (with the value to meet their personal, social, aesthetic, and other needs), compatibility (in line with their characteristics and needs in different periods), and timeliness.

Educators are more likely to upload teaching plans or learning materials related to theoretical education through the network platform, focusing on theoretical indoctrination. However, psychological education, legal education, and life service are relatively few, accounting for only about 30 percent. The content structure is unbalanced, the format and column setting are a little taken for granted, the life, emotion, psychology and other aspects of college students are not enough attention, insufficient guidance, cannot timely and effectively help college students to correctly deal with psychological problems, rational response to emotional fluctuations, and answer the doubts in life. In the survey, more than 70% of the respondents do not often browse the IPE network platform of the school. More than 50% of the respondents just listen to the online class of IPE. The reasons are shown in Figure 9. Among them, 47.12% think the content of network platform is too much political theory, 35.95% are not interested in it, and 22.18% think the update speed is slow. Contemporary college students rely heavily on the Internet and do not like empty, general, and very serious theoretical knowledge. They are more receptive to novel, highly entertaining, and stimulating information. However, the political theory of network carrier content is too strong, which is easy to make college students antipathy.

The article "Research on the Implementation Path of Ideological and Political Education in Private Colleges and Universities under the Network Environment" was retracted in 2023. Reasons: signs of a paper mill; suspected computer-generated content; unreliable results or conclusions; lack of ethics approval or compliance.

### 3.3. Analysis on the Causes of the Existing Problems in the Application of Network in College Students' IPE

As the “fourth media” following newspapers, radio, and television, the Internet can integrate the advantages of traditional media with its unique characteristics of massive information, immediacy of communication, and equality of interaction so as to expand the coverage of education and enhance the interest, affinity, and appeal. It has strong circulation interaction function, infiltration guidance function, cohesion and excitation function, and radiation infection function.

Most of the college students are the “post-2000” generation who grow up together with network technology, and their life and behavior are full of obvious digital and network survival logic. In terms of the way of thinking, they are self-conscious, have a broad vision, flexible, easy to accept new things, and pursue individuality and innovation. In terms of cognition, they pursue diversity and yearn for equal interaction and communication in terms of information acquisition. The cognitive approach is no longer satisfied with the traditional didactic approach and has shifted from external authority to internal processing. In terms of value orientation, they tend to be diversified and have strong tolerance to different values.

There are laws and regulations to follow in cyberspace as in the real world. The carrier supervision of campus network is a complex system, which covers the monitoring of carrier content, the research and judgment of sensitive information, the control, disposal and feedback of harmful content, and so on. The supervision of virtual space needs to increase manpower input, but it cannot be completed by manpower alone. In view of the current situation, there are still hard wounds in the supervision of network carriers in colleges and universities. Next, we need to continue to overcome difficulties so as to nip in the back, master the initiative of carrier regulation, and ensure the safety and reliability of network carrier operation.

## 4. Result Analysis and Discussion

### 4.1. Highlight the Dominant Content of IPE in Private Colleges under the Network Environment

College students should strengthen their recognition of mainstream ideology. The ideological foundation of “two maintenance” is lay down. Any group needs the right leadership. If there is no head teacher's leadership in a class, there will be no cohesion and unity in the class. In addition, class teachers should also guide students to comprehensively study various policies. This is the valuable experience our party has gained from practice and a fundamental guarantee for realizing the Chinese Dream. As a new person of the times, we should highly identify, firmly maintain, and consciously obey them.

The article "Research on the Implementation Path of Ideological and Political Education in Private Colleges and Universities under the Network Environment" was retracted in 2023. Reasons: signs of a paper mill; suspected computer-generated content; unreliable results or conclusions; lack of ethics approval or compliance.

### 4.2. Strengthening the Basic Content of IPE in Private Colleges under the Network Environment

What are the contents of ideological literacy education in colleges and universities under the network? First, carry out education in ideals and beliefs. Ideal is like climbing to the top of the mountain, and faith is the power to support the summit. Ideals and beliefs together constitute ideal beliefs. First of all, General Secretary Xi stressed: “We should use new media and technology to make our work come alive, promote the integration of traditional advantages of ideological and political work with information technology, and enhance the sense of the times and appeal.” Universities should pay attention to students' dynamics, help students build noble character, and enable them to achieve comprehensive and free development. Then, the content of ideal and belief education should be optimized based on realistic needs. Set up with interesting ideological and political theory content so as to firm up their ideals and beliefs.

Secondly, in the face of diversified cultures on the Internet, it is the only way to educate college students on “three views” in order to prevent negative information from affecting their “three views.” First, use a good, healthy culture to take the online ground. Constantly innovate the form of network information dissemination, using the way that college students like to spread ideological and moral theory; use vivid language and typical examples to explain beliefs and integrate boring theoretical content into pictures and animations to improve educational effects. Secondly, the social hot spots of positive energy are used to influence students' “three views.” For example, “The Road of Cultural Creation in the Forbidden City” and “Kang Xi feels cute” are popular online searches. Through this social hot spot, students can feel the excellent culture and form the correct “three views” unconsciously.

Good moral cultivation is the guide to adjust various social contradictions. First of all, society, school, and family should unite to strengthen social moral education. On the one hand, schools should incorporate social morality education into the teaching system, teach relevant theoretical knowledge, and organize relevant practical activities. On the other hand, parents should set an example and pay attention to their words and deeds in daily life, such as showing filial piety to the elderly, caring for children, protecting the environment, and so on. Create comfortable, good family environment; lead students to form good moral quality. We should set up the concept of “great political thinking,” integrate moral education into other education, expand students' thinking breadth, increase the interest of theoretical knowledge, and stimulate students' learning enthusiasm.

The article "Research on the Implementation Path of Ideological and Political Education in Private Colleges and Universities under the Network Environment" was retracted in 2023. Reasons: signs of a paper mill; suspected computer-generated content; unreliable results or conclusions; lack of ethics approval or compliance.

Nowadays, the Internet has become an irreplaceable tool for work and study, bringing new opportunities for college students to improve their cultural literacy. However, the culture on the network is uneven, which requires universities to carry out cultural literacy education based on the network and guide college students to learn excellent cultural knowledge.

First, carry out cultural confidence education. Cultivating a new generation of young people with strong cultural confidence is key if a country or nation wants to develop. In today's society, the lack of culture is becoming more and more prominent. Faced with this situation, we must solve the problem from the root. First, cultivate college students' cultural confidence. Universities should set up courses of traditional culture and encourage students to read relevant books so that students can deeply understand the connotation and essence of Chinese traditional culture. Second, we should stimulate cultural confidence and vitality through cultural innovation. In other words, we should attach importance to cultural innovation, which requires colleges and universities to guide students to base themselves on practice, encourage them to participate in social practice activities, broaden their horizons, increase their understanding of real life, and enable them to carry out cultural innovation better.

Second, regarding traditional culture education, Chinese traditional culture, the soul of our nation, contains rich educational resources. As a place to cultivate new people in the socialist era, colleges and universities must strive to improve students' comprehensive cultural accomplishment. First of all, innovate cultural communication channels. Through classroom, practice, network, and other ways to carry out traditional culture education, enrich the channels of education, expand the coverage of cultural edification, and realize the function of excellent culture in shaping the personality of college students. Secondly, promote the new thinking of traditional culture education. Teachers must change their educational thinking, hand over the classroom to students, and stimulate students' learning enthusiasm.

The article "Research on the Implementation Path of Ideological and Political Education in Private Colleges and Universities under the Network Environment" was retracted in 2023. Reasons: signs of a paper mill; suspected computer-generated content; unreliable results or conclusions; lack of ethics approval or compliance.

Third, carry out advanced cultural education. First, educate students to be leaders of advanced culture. The openness and concealment of network make college students deviate from the direction of advanced culture. Under the complex and diverse cultural background, whether college students can deeply understand the cultural connotation is related to the future era of our country. Therefore, it is necessary to help college students consciously lead the advanced Chinese culture, to deeply exude admiration and pride of Chinese culture from their hearts, and to firm up the belief of excellent Chinese culture from their hearts. Second, educate students to be the inheritors of excellent culture. Whether human society can develop in a civilized and harmonious way is closely related to the function of excellent traditional culture. For example, after the outbreak of COVID-19, the self-discipline of everyone wearing masks, the dedication of staff to stick to their posts, and the friendship of everyone making donations to Wuhan have all formed a strong spirit of epidemic prevention. Obviously, these spirits are the embodiment of the power of Chinese culture. As a college student, we should cherish the learning platform provided by the school, cherish the precious learning time and resources, strengthen the study of excellent cultural knowledge, improve cultural literacy, and firm cultural confidence.

Finally, students are taught to make full use of various practical activities for cultural innovation. Practice is the source of knowledge and the only way to innovate. Universities should encourage more participation in practice.

### 4.3. Increase the Charm of IPE Content in the Network Environment

If we can effectively enhance the attractiveness of the content of the network carrier, it will be conducive to effectively play the educational function of the network carrier. We should adhere to the unification of propagating mainstream culture and advocating cultural diversity, take care of the complexity of college students, improve the truth, value, and reality of carrier content, and enhance the persuasiveness of carrier content communication. As mentioned above, college students have formed the consumption habit of short and quick content and pay little attention to and are not interested in the content of the network carrier of colleges and universities, and there is a certain degree of dislocation between the content of the network carrier and the cognitive structure of college students. For this, we need to organize professional personnel to strengthen team building. We should focus on educating all personnel and promote the building of various specialized teams.

The article "Research on the Implementation Path of Ideological and Political Education in Private Colleges and Universities under the Network Environment" was retracted in 2023. Reasons: signs of a paper mill; suspected computer-generated content; unreliable results or conclusions; lack of ethics approval or compliance.

First, it is necessary to set up a leading team, set up a special organization and leadership organization, unite the publicity department and the student work department, make clear the overall goal, overall planning, and work deployment of the network carrier, and ensure the orderly development of daily work. Second, in terms of education courses, class teachers, teachers, students, and college student party members and cadres should work together to select educators with high ideological and political quality, familiar with the characteristics of network language, and able to skillfully use network carriers. They can also choose top students of different grades, different subject backgrounds, and different majors to form a carrier content planning team. I was responsible for investigating the actual situation of college students on campus, understanding the hot topics of college students, and then making and updating carrier content scientifically, and organizing creative activities with the help of network carrier. Third, to organize review and comment team, the whole network monitoring of carrier content can be carried out, and regularly evaluate feedback, timely find problems, and formulate rectification plan. Secondly, we should strengthen the appeal of network carrier content creation. We should adhere to the theory with practice, through the history and reality in the theoretical discussion, really explain the theory thoroughly, get rid of the formal barriers of abstract theoretical study, achieve convincing people with reason, and let the theory into the mind and heart. Therefore, we should attach importance to the combination of historical events, social events, and practical examples around college students to analyze and interpret scientific thoughts.

Young college students have always been concerned about current affairs, we should assist college students to correctly understand the times and deepen the theoretical cognition. In addition, there are a lot of fresh educational resources around college students. Educational celebrities, academic masters, and peer models are key boosters to guide college students to be good. Campus, dormitory, and family are all important sources of carrier content innovation. We should be close to students' lives and incorporate the vivid materials they have personally experienced and experienced into carrier content to carry forward good fashion. While creating their own content, they can also introduce other excellent network cultural works. It not only includes academic planning, career planning, example demonstration, and theoretical education, but also includes social hot spot analysis, cultural inheritance, and warning education to enrich carrier content and realize value guidance.

The article "Research on the Implementation Path of Ideological and Political Education in Private Colleges and Universities under the Network Environment" was retracted in 2023. Reasons: signs of a paper mill; suspected computer-generated content; unreliable results or conclusions; lack of ethics approval or compliance.

Finally, the practicability of network carrier content design should be improved because the theme that can attract people and be easy to spread is the basic requirement to grasp the attention of college students. Many college students are “clickbait.” They read the headlines before deciding whether to read the content. We should grasp the needs of the times and the general trend of development, dig into various social phenomena, understand the common problems that netizens are concerned about and the individual problems that college students are concerned about. “With a high degree of sensitivity and profound insight, we should distinguish between hot spots and key points, mainstream and tributary, phenomenon and essence, major events and the general trend.” Carefully craft eye-catching issues. At the same time, “seize the opportunity, grasp the rhythm, pay attention to strategy, from the timing of efficiency, and reflect the timing of efficiency requirements.” In addition to the title, sometimes the quality of the cover can directly affect the click-through rate. Therefore, in the cover design, it is necessary to combine the content style to design the cover size reasonably, choose the right template, tone, illustration, entry, and so on, and form a characteristic mode. To set up the content structure reasonably, highlight the original school. While spreading political theoretical knowledge, class teachers should give college students life guidance and psychological guidance, transmit information directly related to their lives, and arouse their interest and attention. In terms of discourse expression, deep feelings should be integrated, and academic language should be combined with life language. Absorb popular words or newly created vocabulary resources in network discourse, integrate symbols and other forms of expression, and shorten the distance with language and diversified expressions that college students can understand. Illustrate the truth with typical examples that are close to life and instructive.

### 4.4. Improve the Supervision System of IPE Practice in the Network Environment

We should improve the management rules and regulations of campus network operators. At present, there are loopholes in the management of network carriers. The competent education department should further interpret the spirit of the policy, implement laws and regulations, and conduct extensive research on the operation and management of network carriers in colleges and universities, so as to comprehensively grasp it and formulate universally applicable guiding norms. We can choose good use cases in network carrier management, summarize experience, promote use, and provide effective communication and collaborative development platform for colleges and universities.

The article "Research on the Implementation Path of Ideological and Political Education in Private Colleges and Universities under the Network Environment" was retracted in 2023. Reasons: signs of a paper mill; suspected computer-generated content; unreliable results or conclusions; lack of ethics approval or compliance.

Colleges and universities should abide by laws and regulations, implement the instructions of competent authorities, and strengthen the publicity of law. It is necessary to define the level and scope of security management, standardize the procedures for using network carriers, maintenance systems, and emergency measures and procedures for handling online disputes, implement the real-name online system, and supervise and control user registration, login, and information release. In addition, some colleges and universities do not have a very perfect evaluation system; there are some problems, such as disordered evaluation target positioning, one-sided evaluation target, formalization, uncertain evaluation range, chaotic evaluation content, single evaluation method, and failure of evaluation guidance and incentive function. Therefore, efforts should be made to improve the evaluation mechanism. First, it is necessary to set up scientific evaluation thoughts, fully understand and absorb the latest educational evaluation theoretical achievements, speed up the transformation of evaluation ideas, and correctly understand the guidance, appraisal, incentive, and adjustment functions of evaluation work. Second, it is necessary to establish a three-dimensional and cross evaluation mechanism, and make comprehensive evaluation through education departments, responsible departments of colleges and universities, educators and recipients, and social evaluation institutions.

Second, perfect the campus network carrier supervision department. To build China into a cyber power, the state has set up the Cyberspace Affairs Commission of the CPC Central Committee, and governments at all levels have information cybersecurity supervision departments. To implement effective supervision, colleges and universities also need to set up special supervision departments, such as network carrier construction department, network carrier application information feedback center, quantitative analysis center, and so on. Full-time personnel are responsible for technology research and development, key management, permission setting, information release, risk assessment, and troubleshooting. Build campus network defense system on the basis of the popularization of campus network, maintain the system regularly, audit the content in the network carrier, and filter spam and illegal information, harassment information, and virus links. The high standard of network supervision for technology needs the support of high-level network security talents. Therefore, colleges and universities need to improve talent training specifications, optimize talent introduction policies, set up relevant specialties and research institutions, hold relevant training, and fill the talent gap.

The article "Research on the Implementation Path of Ideological and Political Education in Private Colleges and Universities under the Network Environment" was retracted in 2023. Reasons: signs of a paper mill; suspected computer-generated content; unreliable results or conclusions; lack of ethics approval or compliance.

Third, strengthen students' sense of self-discipline and enhance their ability of independent supervision. China had 989 million Internet users in 2020, and college students are a more active part of the nearly one billion Internet users. In the campus network carrier supervision, the main body of college students also plays an immeasurable role. Colleges and universities should strive to create a legalized and civilized campus environment, strengthen the publicity of law popularization and cultivation of network morality through classes, lectures, forums, knowledge competitions, campus banners, micro films, and other ways, and guide students to enhance network self-discipline and establish correct network cognition. College students should also consciously improve the network ideological and moral cultivation, self-examination and self-correction, and self-restraint. Think deeply and independently before speaking, and avoid stereotypes. Do not make assumptions about hot issues. Do not engage in personal attacks when sharing ideas. To the emergency to investigate the truth, do not forward comments at will, the formation of false induction. Strengthen the awareness of network security, establish the concept of network law, consciously abide by laws and regulations, to achieve online self-discipline, self-examination, and self-protection. Be alert to audio, video, and written remarks containing extremism, separatism, and terrorism on the Internet; report them immediately and stop watching them once found. Do not comment, do not discuss, do not take the initiative to download and save relevant materials, do not forward and spread, and improve sensitivity and insight. In addition, the school can try to establish a student volunteer team, can also allocate some funds for students to work and study, and participate in the monitoring and maintenance of the campus network carrier. Students can also be regularly organized to conduct a questionnaire survey or interview, self-evaluation, reflection on their own thoughts, cognition and behavior, and combined with praise, reward, and other ways to encourage students to self-monitoring. We should also attach importance to all kinds of student organization resources, and they should take the lead in organizing propaganda and education activities and mobilizing college students to participate in network supervision. In a word, college students should play the main role, pay close attention to the network information, monitor the content of the network carrier, enhance the awareness of prevention, improve the screening ability, and timely find, report, and deal with bad information. To improve the rules and regulations, manage kinds of processes and other valuable suggestions.

The article "Research on the Implementation Path of Ideological and Political Education in Private Colleges and Universities under the Network Environment" was retracted in 2023. Reasons: signs of a paper mill; suspected computer-generated content; unreliable results or conclusions; lack of ethics approval or compliance.

## 5. Conclusion

In the era of “Internet + education,” the Internet has become the main way for private college students to directly obtain information. Private colleges and universities should only build a “network ideological and political” pattern under the unified leadership of the party committee, and build a main force of network ideological and political construction with excellent ability and quality. Therefore, this paper firstly elaborates the concept of PCU, introduces the current situation of IPE of students in PCU in China under the network environment, and studies the corresponding countermeasures and the paths of subsequent practice through the research and analysis of existing problems. There is still a lot of space for the research on IPE of college students in the network environment, and in the future, the author will conduct deeper research on the IPE of students in PCU in China in the network environment. On the basis of the original research, further attempts will be made to find a new construction path.

## Figures and Tables

**Figure 1:** Internet users and internet penetration.

**Figure 2:** Age structure.

**Figure 3:** Education structure.

**Figure 4:** Age distribution.

**Figure 5:** Education level.

**Figure 6:** Application effect of IPE network carrier.

**Figure 7:** Teachers' proficiency in using network carriers.

**Figure 8:** Frequency of communication between teachers and counsellors and students through the network platform.

**Figure 9:** Reasons for infrequent browsing of IPE network platforms.

**Table 1:** The impact of internet.

Added learning materials (%)	Changed the way of learning (%)	Broaden the scope of knowledge (%)	Conducive to professional learning (%)	No impact on study (%)	Interfered with normal study (%)
75.50	38.60	81.70	85.80	11.90	4.20

**Table 2:** The impact of Internet access on college students' interpersonal communication.

Made new friends through the Internet (%)	Keep in touch with netizens (%)	Wants to try online dating (%)	Making friends online affects daily communication (%)	Do not want to make friends through the Internet (%)
61.5	49.5	49.7	38.6	1.1

The article "Research on the Implementation Path of Ideological and Political Education in Private Colleges and Universities under the Network Environment" was retracted in 2023. Reasons: signs of a paper mill; suspected computer-generated content; unreliable results or conclusions; lack of ethics approval or compliance.

**Table 3:** Proportion of young netizens agreeing with the view that “if you do not surf the internet for a day, you feel you lack something.”

Nonstudents (%)	College student (%)	Primary and secondary school students (%)	Youth Internet users in general (%)	National Internet users (%)
36.5	26.8	21.0	27.1	38.3

**Table 4:** Main activities of students on the Internet.

Options	Subtotal	Proportion
Internet chat	255	63.75%
Watch videos and listen to music	288	72.00%
Watch news	116	29.00%
Find study materials	208	52.00%
Find information about life (shopping, etc.)	93	23.25%
Browsing posting, forums, knowledge, personal web pages, etc.	90	22.50%
Online games	36	9.00%
The number of people who filled in this questionnaire is valid	400	—

## Data Availability

The labeled dataset used to support the findings of this study are available from the corresponding author upon request.
